# A Convolutional Neural Network Algorithm for the Optimization of Emergency Nursing Rescue Efficiency for Critical Patients

This article has been retracted.

**DOI:** 10.1155/2021/1034972

**Published:** 2021-10-06

**Authors:** Xueyan Chen, Xiaofei Zhong

**Affiliations:** ^1^Emergency Department, Zhejiang Hospital, Hangzhou, Zhejiang 310030, China; ^2^Neurosurgery Department, Zhejiang Hospital, Hangzhou, Zhejiang 310030, China

## Abstract

In order to help pathologists quickly locate the lesion area, improve the diagnostic efficiency, and reduce missed diagnosis, a convolutional neural network algorithm for the optimization of emergency nursing rescue efficiency of critical patients was proposed. Specifically, three convolution layers and convolution kernels of different sizes are used to extract the features of patients' posture behavior, and the classifier of patients' posture behavior recognition system is used to learn the feature information by capturing the nonlinear relationship between the features to achieve accurate classification. By testing the accuracy of patient posture behavior feature extraction, the recognition rate of a certain action, and the average recognition rate of all actions in the patient body behavior recognition system, it is proved that the convolution neural network algorithm can greatly improve the efficiency of emergency nursing. The algorithm is applied to the patient posture behavior detection system, so as to realize the identification and monitoring of patients and improve the level of intelligent medical care. Finally, the open source framework platform is used to test the patient behavior detection system. The experimental results show that the larger the test data set is, the higher the accuracy of patient posture behavior feature extraction is, and the average recognition rate of patient posture behavior category is 97.6%, thus verifying the effectiveness and correctness of the system, to prove that the convolutional neural network algorithm has a very large improvement of emergency nursing rescue efficiency.

## 1. Introduction

Pathological diagnosis plays an important role in the diagnosis and treatment of diseases. Pathologists have the reputation of “doctors' doctors.” 70% of medical diagnosis depends on pathological diagnosis, which is considered as the “gold standard” of disease diagnosis. However, there are many problems in the pathology industry. There is a huge shortage of pathologists in China, and there are only about 20,000 pathologists in China [1]. It is difficult to train pathologists. A pathologist needs to cover the diagnosis of each system of the human body and memorize the morphology of more than 15 000 pathological samples and more than 5 000 basic disease names. It takes more than 10 years to train a mature pathologist, and it is difficult to fill the gap in the short term. Pathologists have a heavy workload, with up to 150 cases of difficult pathological diagnosis in and out of the hospital every day [2]. There are regional differences in pathological medical resources. 70% of pathologists in China are concentrated in level-III hospitals, while there are more than 20,000 level-II and below hospitals with only 0.12 pathologists in each hospital on average, which cannot meet a large number of clinical pathological diagnosis needs of primary hospitals. Artificial intelligence technology is used to enable digital pathological diagnosis. Through training and learning massive confirmed pathological images, intelligent recognition of pathological images can be realized quickly, thus greatly improving the efficiency and accuracy of pathological diagnosis. Valova et al. proposed to use experience to improve the performance of the system itself by means of calculation. Reinforcement learning is to interact with the environment, judge the next action according to the reinforcement signal provided by the environment, and constantly improve the action plan to adapt to the current environment. In recent years, machine learning algorithms have been widely used in disease prediction (heart disease, diabetes, breast cancer, thyroid, etc.) [3]. Chang et al. proposed to use convolutional neural network algorithm to predict heart disease. Firstly, data information such as user's age, gender, blood pressure, heart rate, cholesterol, diabetes, and obesity were collected. Secondly, a machine learning model to predict heart disease was constructed by using multilayer perceptron neural network structure; the multilayer perceptron model has simple structure and high efficiency and is generally suitable for processing data sets with small data dimensions. Mmnmayi et al. proposed to use support vector mechanism to build a disease prediction model, which is to use datasets in daily life to predict diseases frequently occurring in daily life. Support vector machine is suitable for processing high-dimensional data, but it has the problem of high computational complexity, and the accuracy of disease prediction model constructed by support vector machine algorithm needs to be further improved [4]. Cheng et al. proposed using three algorithms of support vector machine, Bayesian network, and decision tree to predict diabetes and introduced principal component analysis on this basis to carry out dimension-reduction processing on data [5]. On the basis of the current research, this paper uses three convolutional layers with different sizes of convolution kernel to extract the patient's body behavior features. The classifier of the patient's body behavior recognition system learns the feature information by capturing the nonlinear relationship between features, in order to achieve accurate classification, the accuracy of the patient's body behavior feature extraction network, the recognition rate of a certain action, and the average recognition rate of all actions in the patient's body behavior recognition system, to prove that the convolutional neural network algorithm has greatly improved the efficiency of emergency nursing rescue [6].

## 2. Methods

Research on patient posture behavior recognition technology based on convolutional neural network; there are three main problems; firstly, the individual difference and nonrigid deformation of patients bring great difficulty to the detection of body posture behavior. Secondly, multiperson scenes and complex backgrounds will also affect the detection, and the real-time and reliability of the detection and identification system cannot be guaranteed [7]. Finally, the diversity of perspectives, a variety of human posture, monitoring probe shooting angle, is not the same, which also brings great challenges to patient detection. Convolutional neural network is a kind of feedforward neural network, which is specially used to process data with grid structure such as image. In order to solve the goal of detecting patient posture behavior in intelligent medical care, the convolutional neural network structure and training label are designed, and the algorithm of detecting patient posture behavior is proposed. Finally, the proposed algorithm is verified and analyzed. The convolutional layer is the core of the convolutional neural network, which extracts features from the input layer. The excitation layer makes a nonlinear mapping of the output results of the convolution layer [8]. The pooling layer is mainly responsible for compressing the amount of data and parameters to avoid overfitting. The full connection layer is located at the tail of the convolutional neural network, which has the same connection mode as the traditional neural network. In the research of intelligent medical care based on convolutional neural network, a dual network model is adopted. Firstly, a patient detection network model is designed, and then, a patient body motion feature extraction network model is designed. In the research of intelligent medical care based on convolutional neural network, a dual network model is adopted. Firstly, a patient detection network model is designed, and then, a patient body motion feature extraction network model is designed. Patient detection is a detection mechanism that uses a target detection algorithm to determine the target position. By combining target detection with patient posture behavior feature extraction, the target patient can be better targeted and then the patient's posture behavior feature can be recognized [9]. YOLO algorithm is based on deep learning target detection algorithm. YOLO algorithm can detect the position of target bounding box quickly, efficiently, and accurately and in real time. In the YOLO algorithm, the input image is divided into *n* × *n* square grids to determine whether the center of the target object falls inside the grid. If so, the grid is marked to represent that the grid can detect the target object. For each cell, *m* bounding boxes and the confidence of the bounding boxes can be predicted:

(1) $$\begin{array}{c} C=\mathrm{Pr}\left(\text{object}\right)*LOU_{\text{pred}}^{\text{truth}}, \end{array}$$

where Pr(Object) represents the probability that the bounding box contains detecting targets and *LOU*_pred_^truth^ represents the accuracy of the bounding box.

(*x*, *y*, *w*, *h*) is used to represent the size and position of the bounding box, where (*x*, *y*) represents the center coordinate of the bounding box, and *w* and *h* represent the width and height of the bounding box. Therefore, the predicted value of the bounding box is (*x*, *y*, *w*, *h*, *c*). *K* class probability value is given for each grid; the probability value is the conditional probability under Pr (object), notes for Pr (class_*i* | object). Thus, the category confidence of the bounding box is defined as

(2) $$\begin{array}{c} \mathrm{Pr}\left({\text{class}}_{i}|\text{objiect}\right)*\mathrm{Pr}\left(\text{object}\right)*IOU_{\text{pred}}^{\text{truth}}=\mathrm{Pr}\left({\text{class}}_{i}\right)*IOU_{\text{pred}}^{\text{truth}}. \end{array}$$

According to the above research and analysis, the YOLO algorithm is obtained as follows.

Input: an image of 448 × 448 pixels. Output: a result vector representing the category, size, and position of the bounding box. Step 1: enter the required detection image. Step 2: split the target image into a *n* × *n* grid step to determine that the object center is in the no grid. If so, enter Step 3. If no, go to step 9. Step 3: forecast *m* target boundaries using the grid. Step 4: calculate the central coordinates of the target boundary frame, wide, high, and confidence vectors (*x*,. *y*, *w*, *h*, *c*). Step 5: prediction of a category Pr (class_*i* | object). Step 6: calculate bounding box category confidence using formula (2). Step 7: eliminate redundancy with nonmaximum suppression algorithm. Step 8: algorithm outputs the most accurate and effective bounding box result first vector. The patient body movement feature extraction network model uses YOLO algorithm to detect and locate the patient and then uses the patient body movement feature extraction network model to extract the patient feature information [10]. A convolutional neural network with three convolutional layers of different sizes is proposed to extract the body behavior characteristics of patients simultaneously. The size of the convolution kernel affects the size of the local receptive field. The size of the convolution kernel is generally smaller than the size of the input image, and the features extracted by the convolution will emphasize more on local features, which is very consistent with the image processing we are exposed to in daily life. In the real scene, each neuron does not need to perceive the global image. Instead, it senses the local features and synthesizes the local information at a higher level so as to obtain the global information. The size of the traditional convolution kernel is all set to an odd number. For example, the size of the 3 × 3 convolution kernel affects the size of the local receptive field. The size of the convolution kernel is generally smaller than the size of the input image, and the features extracted by the convolution will emphasize more on local features, which is very consistent with the image processing we are exposed to in daily life. In the real scene, each neuron does not need to perceive the global image, but perceives the local features and synthesizes the local information at a higher level to obtain the global information [11]. Traditional convolution kernel sizes are all set to odd numbers, such as 3 × 3, 5 × 5, or 7 × 7. The reason why the size of the convolution kernel is chosen as an odd number is because of the following potential advantages. Protecting the position information: the “anchor point” is just in the middle, which is convenient for sliding convolution based on the center of the module and avoids the “offset” of position information. In view of these problems, the basic unit in the model was improved, and three convolutional layers with different sizes of convolutional kernel were used to extract the patient's body behavior characteristics. The inception improved model is shown in Figure 1.

In the structure model of body feature extraction network, 30 new feature maps are obtained from input data through the first inception structure. After the second and third inception structures, 90 and 270 feature patterns are obtained, respectively. There is no convolutional layer of 3 × 3 convolutional core in the structure. How can the convolution layer of 3 × 3 convolutional core be finally output? Then, the body behavior characteristics of patients are extracted through the convolutional layer of two 5 × 5 convolutional kernels. Finally, output through the convolution layer of 7 × 7 convolution kernel. After designing the network structure, the classifier should be designed for the patient posture behavior algorithm. When the patient posture behavior features are extracted, the recognition results of the patient posture behavior categories are given according to the classifier. The global average pooling layer and Softmax layer are used as the classifier. When the data in the dataset are processed once by the constructed model and returns once, the process is called one iteration. However, in the whole experiment, if only one EPOCH is set, the computer will have a heavy load, a heavy computing burden, and a slow running speed. Therefore, all datasets need to be processed into blocks; the complete dataset is transmitted in the same neural network for many times. With the increase of the number of epoch, the updating times of weights in the neural network are also increasing, and the network model is easily changed from underfitting to overfitting. The experimental results show that the size of EPOCH has a great influence on the accuracy of the model. If the epoch is too small, the model will have insufficient learning ability, large deviation, and insufficient learning and training, resulting in a low accuracy of the model [12]. If the epoch is too large, the model will tend to converge after a certain number of iterations, which will not only fail to improve the correct recognition rate but also increase the training time of the model and may even cause the problem of overfitting. In this way, the network parameters of the identification system can be reduced to ensure the efficient operation of the system. The classifier of the patient's body behavior recognition system is shown in Figure 2.

Among them, the main role of the GlobaoAveragePooling layer is to pool and reduce the dimension of feature map, while the main task of Softmax layer is to output the final result with probability. Usually, there are multiple types of feature subgraphs, each of which is composed of some neurons arranged in a rectangular form, and the weight parameters among the neurons are shared. This approach can significantly reduce the connections between all layers of the network, thus reducing network parameters, and at the same time avoid overfitting [13]. In the neurons of the neural network, the neurons will be activated only when the weighted sum value of the signals of the neurons in the current layer is greater than the artificially fixed threshold value, that is, the activation function is used to determine whether the output of each neuron exceeds the threshold value. In the convolutional neural network, if the feature strength of a specific region does not reach a certain standard, 0 will be output, indicating that the feature of this region is very weak and cannot be extracted from this region. When output 0, the gradient of the activation function is basically close to 0, so in the area with weak features, the gradient will not decrease basically, that is, the area unrelated to this feature will not affect the extraction of other features by this training [14]. Therefore, the nonlinear activation function can significantly reduce the influence of irrelevant features. In convolutional neural networks, nonlinear functions are usually used as activation functions to improve the expression ability of models. Subsampling, also known as pooling, can be regarded as a special convolution process. The convolution process and subsampling can greatly reduce the parameters of the model and simplify the complexity of the model. Subsampling usually has two forms: mean subsampling and maximum subsampling. It can reduce the error caused by the increase of the variance of the estimated value caused by the neighborhood size limitation and retain more background information of the image. The error caused by the deviation of the estimated mean value caused by the parameter error of the convolutional layer is reduced, and more texture information is retained. It is worth mentioning that the function of the maximum subsample operation is that, as long as a feature is extracted, it will remain in the maximum subsample output. Therefore, the practical function of the maximizing subsampling operation is that if a feature is extracted from the convolution kernel, the maximum value is retained [15]. If this feature is not extracted, it may not exist, or the feature is not obvious; then, the maximum value of the region is still very small. Therefore, the experimental results of maximum subsampling are very good. Data features go through several steps such as convolution calculation and subsampling calculation. Before output, they have to go through the full connection layer; the purpose of the full connection layer is to map the feature information learned in the convolutional neural network to the label space of the sample. After the processing of the full connection layer, the two-dimensional feature map outputs after the convolution processing will be transformed into a one-dimensional feature vector, which is to synthesize all the previously extracted feature information [16]. Then, the whole neural network training is carried out through *N* layers of hidden layers. Compared with the convolutional computing layer, every neuron node in the full connection layer is connected with all the neuron nodes in the upper layer. When the full connection layer acts, the feature information extracted from the convolutional layer is integrated, and the feature information is learned by capturing the nonlinear relationship between features, so as to achieve accurate classification.

## 3. Results and Analysis

Experimental verification of the proposed algorithm was carried out. First, open source framework platforms, Darknet and Caffe, were built to conduct patient detection training and extraction of patient posture and behavior features [17]. Then, the intelligent medical care system based on convolutional neural network is tested. In the test process, 100,000 images of patient detection dataset are prepared, and 50,000 images of network dataset are extracted from body posture behavior characteristics. Finally, the two datasets are divided into two parts: training set and test set, which are, respectively, run on two framework platforms.  Figure 3 shows the accuracy of the patient posture behavior feature extraction network [18].

Table 1 shows the recognition rate of a certain movement and the average recognition rate of all movements in the patient posture behavior recognition system.

The characteristic of convolutional neural network is that convolutional neural network introduces the concepts of weight sharing (convolutional kernel) and receptive field, which greatly reduces the number of parameters that the network needs to learn; the convolutional neural network can reduce the amount of calculation and save the time of calculation and has stronger learning ability and computing power [19]. Improve the efficiency of emergency nursing and rescue.

## 4. Conclusions

This research mainly studies the application of convolutional neural network in image recognition and connects image recognition with intelligent medical care. By proposing a convolutional neural network-based patient posture behavior feature extraction algorithm, the algorithm adopts dual network model design, including the patient detection network model and the patient posture behavior feature extraction model. The algorithm is applied to the patient posture behavior detection system, so as to realize the identification and monitoring of patients and improve the efficiency of emergency nursing rescue. By using three convolutional layers of different sizes of the convolution kernel to extract the patient's body behavior features, the classifier of the patient's body behavior recognition system learns the feature information by capturing the nonlinear relationship between features, in order to achieve accurate classification, the accuracy of the patient's body behavior feature extraction network, the recognition rate of a certain action in the patient's body behavior recognition system, and the average recognition rate of all actions, to prove that the convolutional neural network algorithm has a great improvement in emergency nursing rescue efficiency. In health-related businesses, this paper extracts the characteristics of the patient by three layers with different convolutional cores, learns the characteristics, realizes the precise classification and the accuracy of the network, and proves the efficiency of emergency care. The algorithm is applied to the patient behavior detection system to identify and monitor patients and improve the level of intelligent medical care. The greater the test data collection, the higher the extraction accuracy of patient state behavior characteristics, and the average recognition rate of patient state behavior categories is 97.6%, thus verifying the effectiveness and correctness of the system, to prove that the convolutional neural network algorithm greatly improves the efficiency of emergency care.[20]

## Figures and Tables

**Figure 1:** Inception improved model.

**Figure 2:** Classifier of the patient body behavior recognition system.

**Figure 3:** Accuracy of patient posture behavior feature extraction network.

**Table 1:** The recognition rate of a certain movement and the average recognition rate of all movements.

Species	Bend over	Kick	Wave	Applause.	Go	Run	Sit	Lying	Standing	Squat down	Fall
Number of samples	930	920	890	800	1010	950	990	860	900	860	890
Identification number	918	894	875	786	987	939	975	825	875	842	874
Recognition rate	98.7	97.2	98.3	98.2	97.7	98.8	98.5	95.9	97.2	97.9	98.2
Average recognition rate	97.9										

## Data Availability

The data used to support the findings of this study are available from the corresponding author upon request.
